# Privacy Preserved Cervical Cancer Detection Using Convolutional Neural Networks Applied to Pap Smear Images

**DOI:** 10.1155/2023/9676206

**Published:** 2023-07-08

**Authors:** Shtwai Alsubai, Abdullah Alqahtani, Mohemmed Sha, Ahmad Almadhor, Sidra Abbas, Huma Mughal, Michal Gregus

**Affiliations:** ^1^College of Computer Engineering and Sciences, Prince Sattam Bin Abdulaziz University, Al-Kharj, Saudi Arabia; ^2^Department of Computer Engineering and Networks, College of Computer and Information Sciences, Jouf University, Sakaka 72388, Saudi Arabia; ^3^Department of Computer Science, COMSATS University, Islamabad, Pakistan; ^4^Department of Computer Science, Kinnaird College for Women, Lahore 54000, Pakistan; ^5^Information Systems Department, Faculty of Management, Comenius University in Bratislava, Odbojárov 10, 82005 Bratislava 25, Slovakia

## Abstract

Image processing has enabled faster and more accurate image classification. It has been of great benefit to the health industry. Manually examining medical images like MRI and X-rays can be very time-consuming, more prone to human error, and way more costly. One such examination is the Pap smear exam, where the cervical cells are examined in laboratory settings to distinguish healthy cervical cells from abnormal cells, thus indicating early signs of cervical cancer. In this paper, we propose a convolutional neural network- (CNN-) based cervical cell classification using the publicly available SIPaKMeD dataset having five cell categories: superficial-intermediate, parabasal, koilocytotic, metaplastic, and dyskeratotic. CNN distinguishes between healthy cervical cells, cells with precancerous abnormalities, and benign cells. Pap smear images were segmented, and a deep CNN using four convolutional layers was applied to the augmented images of cervical cells obtained from Pap smear slides. A simple yet efficient CNN is proposed that yields an accuracy of 0.9113% and can be successfully used to classify cervical cells. A simple architecture that yields a reasonably good accuracy can increase the speed of diagnosis and decrease the response time, reducing the computation cost. Future researchers can build upon this model to improve the model's accuracy to get a faster and more accurate prediction.

## 1. Introduction

Cervical cancer occurs when a cell inside the cervix begins to proliferate rapidly, thus making it a malignant cell. A virus known as human papillomavirus (HPV) is responsible for developing cancerous cells [1]. When detected early, cancer can be treated and rapidly become fatal if ignored. One of the leading causes of mortality in women worldwide is cervical cancer. Women under 30 are at high risk for the disease [2]. According to the Centers for Disease Control and Prevention (CDC), in the US alone, about 13000 women suffer from the disease each year, resulting in around 4000 casualties [3]. Around 604 000 women worldwide were diagnosed with cervical cancer, and 342 000 deaths were reported in 2020 owing to cervical cancer [4]. These alarming numbers have highlighted the need for prompt action to detect, diagnose, treat, and prevent the disease. Detecting the disease in its preinvasive stage shows a promising disease prognosis. Two of the most common techniques to detect the precursor for cervical cancer are the PAP smear and HPV testing [5].

A Pap smear test can be very time-consuming since it requires a radiologist's examination of some 10000 cells to identify any abnormality in cells [6]. For this reason, modern healthcare has turned to artificial intelligence and deep learning to detect and diagnose cervical cancer. Not only can an automated process detect cancer cells in a fraction of the time but it can give objective and accurate results. Researchers have performed image classification on Pap smear test data and analyzed the images to detect abnormalities. A CNN is commonly used for image classification. A CNN can automatically extract features from the image and use it to classify the image as a healthy cell or a cancerous cell. Our proposed CNN model is applied to single cervical cell images and classifies each cell into one of the five categories. An infected cell has different shape, color, and nuclei characteristics. Accurate detection of the nuclei during segmentation can also give a good approximation of the cytoplasm [7]. These features, once extracted, can give an accurate prediction using the CNN model.

The biggest challenge in Pap smear analysis for cervical cancer detection is the complexity and accuracy of the exam. The morphology of cervical cells varies significantly in terms of color, size, and shape [8]. It is difficult to differentiate between different cell types with the naked eye [9]. The primary motivation for developing a CNN model to classify cervical cells was to reduce the complexity and speed of the classification process. Many researchers have attempted to automate this process to achieve more accurate results. It has been observed that high levels of accuracy have been achieved via transfer learning, with complex CNN architectures like the Alex-Net, VGG-net, and ResNet [10–16]. The computational needs of these architectures are tremendous, with longer processing times and requiring a more powerful machine [17]. The ongoing efforts to reduce CNN complexity for cervical cancer detection yield promising results. We aim to create a CNN model that is accurate and computationally efficient.

The paper contributes to the research of automated cervical cancer detection in the following aspects:

- Propose an approach to classify a cervical cell as cancerous or noncancerous by identifying its type from among the five different types
- Expand the data by using data augmentation techniques, giving an excellent generalization to the model
- A combination of different convolutional layers and max-pooling layers have been used to achieve good prediction accuracy
- Achieve promising results with minimum complexity and earliest response time

The rest of the paper is organized as follows: Section 2 presents a literature review of the existing work done by different researchers. We analyzed the current work to find the research gaps in cervical cancer cell detection.  Section 3 elaborates on our proposed methodology, which covers the data selection, data preprocessing techniques used, and a breakdown of our proposed architecture.  Section 4 overviews the experimental analysis and the results obtained using the proposed CNN architecture. The accuracies and the loss comparisons are made in this section.  Section 5 discusses the conclusion of our research.

## 2. Literature Review

Several authors have proposed machine learning and deep learning models for cervical cancer prediction. Research that used Pap smear image data has mainly proposed CNN models and achieved very high accuracy levels. The authors in [6] proposed a model that uses a CNN model to predict cervical cancer by first applying a two-step feature reduction approach. PCA (principal component analysis) was used to reduce the dimensionality of the image data. An optimal feature subset was then obtained using the GWO (grey wolf optimizer). The new optimum feature set improves the classification process. The authors used three famous datasets for training the proposed CNN model: the Mendeley Liquid Based Cytology dataset, the Herlev Pap Smear dataset, and the SIPaKMeD Pap Smear dataset considerably high accuracies for all three datasets. In [18], the author first identified tumor cells by clustering, called the hotspot method. The detected tumor cells were trained using a deep learning model, i.e., a CNN model. Five activation sets were identified, and the best activation set was selected using the pigeon-inspired optimizer. The entire process yielded outstanding results; i.e., 99.6% accuracy was achieved. In another similar work [19], the authors have also proposed a CNN model for detecting and classifying cervical cancer. By analyzing the images of cells via the CNN model, applied to the Herlev dataset, features are learned, and the images are classified using an extreme learning machine- (ELM-) based classifier. Multilayer perceptron (MLP) and autoencoder- (AE-) based classifiers were also used for classification and prediction. The proposed model was able to achieve 99.5% accuracy for detection and 91.2% accuracy for classification of the cell type. [20] is another study that has used six different pretrained CNNs: AlexNet, VGGNet (VGG-16 and VGG-19), ResNet (ResNet-50 and ResNet-101), and GoogLeNet architectures for classification of cells in their precancerous stage and compares their results. An ensemble classifier was then used using the three best models to develop a classifier with excellent accuracy. Hospital-based Pap smear dataset and the Herlev dataset were two data sources used in this model. In [21], the authors have proposed a new CNN model named Colposcopy Ensemble Network (CYGNET) to classify cells using colposcopy images to differentiate between healthy and cancerous cells in the cervix. They have compared and contrasted the results with results obtained on a VGG-19 model used for transfer learning. The proposed model has shown a 19% higher accuracy than the VGG model. The authors of [22] proposed two lightweight CNN architectures for classifying cervical cancer. One model was developed using three convolutional layers, and the other was developed using two convolutional layers with a 2 × 2 stride. ReLU and hyperbolic activation functions have been used to extract features. The models have yielded an area under the curve score of up to 80%.

## 3. Proposed Methodology

Classification of each cell enables accurate and quick detection of malignant cells within the cervix. The proposed work is aimed at classifying cervical cell images into 1 of the five categories, dyskeratotic, koilocytotic, metaplastic, parabasal, and superficial-intermediate, using a CNN. The cell classification identifies cell abnormalities, detecting the precancerous stage and allowing for an early diagnosis to manage disease progression. The proposed work involves data selection, preprocessing and augmentation, model training, and model accuracy.

Figure 1 is the visual representation of how our model works. After performing mathematical operations, the output size increases at each CNN layer, while the max-pooling function reduces the output size by half. The flattened layer makes it easy for the dense layer to connect, reducing the output size to five classes.

### 3.1. Data Selection

Pap smear images are one of the primary methods of cervical cell examination. Several publicly available datasets of Pap smear images containing cluster cervical cell images are available. We use one of the most famous SIPaKMeD datasets. SIPaKMeD represents five cell category names: superficial-intermediate, parabasal, koilocytotic, metaplastic, and dyskeratotic. It contains images of 966 clusters of cell images obtained from Pap smears using CCD camera connected to a microscope. These clusters have been cropped to obtain 4049 individual cell images. It is a labeled dataset where each cropped cell image is classified into one of the five categories. Superficial-intermediate and parabasal are standard cell types; koilocytotic and dyskeratotic cells are those cells that are detected with abnormality but are not malignant. The fifth category of benign cells is classified as metaplastic [23].  Figure 2 is a koilocytotic cell obtained from the dataset. It is marked as abnormal but not malignant. Such cells can indicate precancerous abnormality in the cells. A parabasal cell, a normal cell, appears, as shown in Figure 3.

### 3.2. Data Preprocessing

Image classification requires images to be standardized and scaled.

#### 3.2.1. Image Segmentation

Pap smear slide images were segmented by identifying cells using predefined nuclei and the area of cytoplasm. The border was created around cells of width 1 pixel. The images were then resized to 256 × 256 pixel size.

#### 3.2.2. Categorical Data

The five classes, dyskeratotic, koilocytotic, metaplastic, parabasal, and superficial-intermediate, were assigned five numeric labels: dyskeratotic: 0, koilocytotic: 1, metaplastic: 2, parabasal: 3, and superficial-intermediate: 4.

#### 3.2.3. Data Augmentation

The dataset was expanded by augmenting the images. Four different operations were performed on the training data cell images as shown in Table 1. The training images were augmented using the rescale, flip horizontally, zoom range, and shear range operations. The validation and test data were only rescaled. For training, 2832 cell images were obtained from five classes after data augmentation. 608 cell images were obtained for validation, and 609 cell images were specified for testing.

### 3.3. Proposed Architecture

A CNN is a feed-forward neural network commonly used for image classification. Different layers are applied in the model to classify the data. The proposed classification model is a CNN with 11 layers. Four convolutional layers, three max-pooling layers, three dense layers, and 1 flatten layer have been used to formulate the CNN. Input at the first layer of the CNN model was a 256 × 256 pixel cell. The rectified linear function (ReLU) was applied at all four convolutional layers along with a max-pooling layer of size 2 × 2 to reduce the no. of input parameters to half. The convolutional layer passes extracted feature to the flattened layer. A flattened layer and three fully connected layers in the end help converge the data and are pretty helpful in image classification. A sigmoid function, in the end, returns a binary classification for each of the 5 class outputs.  Figure 4 illustrates the complete architecture of the proposed CNN model.

#### 3.3.1. Convolutional Layer

A convolution layer is the primary component of the CNN model. It extracts features using a combination of convolution operation and activation function [24]. A filter is slid over the input image using a parameter called “stride” that identifies the number of pixels to slide over. The dot product is taken between the filter and the subsection of the input image as per the size of the filter [25]. In our proposed model, 4 convolutional layers were applied using a 3 × 3 filter. The output size/filters for the first two convolutional layers are 32, thus generating 32 output values. The last two convolutional layers generate 64 and 128 outputs, respectively. A ReLU (rectifier linear function) was used to compute the output after each convolution.

#### 3.3.2. Pooling Layer

The pooling layer reduces the size of the extracted feature map that has been processed in the convolutional layer. This is achieved by reducing the connection between layers by selecting just a few pixels from the subsection based on predefined criteria to reduce the computational cost. Hence, pooling can be used for more compact representations while preserving only the most relevant features [26]. Various pooling techniques have been proposed. These techniques are employed based on the different research objectives and desired outcomes, e.g., max pooling, average pooling, sum pooling, soft pooling, stochastic pooling, spatial pooling, and higher-order pooling. The proposed architecture employs a max-pooling layer with a pool size equal to 2 × 2. Thus, after each max-pooling operation, the number of outputs reduces to half the size of inputs. A max-pooling layer was added after each convolution except for the first convolutional layer.

#### 3.3.3. Flatten Layer

The flattened layer is usually placed just before the dense layer to convert the data into a one-dimensional array [27]. This is important to bring the image data into a form that can result in a binary output and be able to classify the image eventually. After all the convolutions were performed, a flattened layer was inserted into the proposed architecture. This has helped convert the 3-dimensional output into a one-dimensional output.

#### 3.3.4. Fully Connected Layer

The fully connected (FC) layer is a combination of the weights, biases, and neurons and acts as a transition to bring it into the desired output form. These layers are usually placed before the output layer and form the last few layers of a CNN architecture. The output of the final fully connected layer has the same number of output nodes as the number of classes [24]. There are three fully connected dense layers at the end of the model. This reduced the output drastically from 115200 (obtained from the flattened layer) to 5 outputs, where each output corresponds to a cell category.

### 3.4. Evaluation Metrics

Several measures have been used to evaluate the performance of our CNN model. The proposed model is assessed based on accuracy, log loss, or categorical cross entropy.

#### 3.4.1. Accuracy

Accuracy is the measure of how well a model performs. It is computed by calculating the no. of correct predictions for a particular class as a ratio of the total no. of predictions. We computed the accuracy of the CNN by calculating the number of correct predictions made by the model for each cervical cell image using the following equation:

(1) $$\begin{array}{c} \frac{\text{TP}+\text{TN}}{\text{TP}+\text{TN}+\text{FP}+\text{FN}}, \end{array}$$

where TP and TN are true positive and true negative, respectively, representing correctly classified cases, and FP and FN are false positive and false negative, respectively, representing the misclassified cases. A value nearer to 1 shows a high level of accuracy achieved.

#### 3.4.2. Categorical Cross Entropy/Log Loss

Cross entropy is the most commonly used loss calculation function in CNNs. The probability of predicted class vs. the actual class output, i.e., 0 or 1, is compared, and a loss is assigned that acts as a penalty in case the predicted value is far from the actual value. This value is a logarithmic value where higher loss means a higher difference in predicted and actual and vice versa. During the training phase, the cross entropy loss is computed and helps adjust weights after each iteration through backpropagation. With each adjustment, the aim is to reduce the loss. The cross entropy of a good model is somewhat close to 0 [28]. Binary cross entropy computes loss for true and false classes, whereas the categorical cross entropy computes the loss for each class and is computed using the following equation [29]:

(2) $$\begin{array}{c} -\frac{1}{N}\overset{N}{\underset{i=1}{\sum }}\overset{C}{\underset{c=1}{\sum }}1_{y_{i}\in C_{c}\log\left(p_{\text{model}}\left[y_{i}\in C_{c}\right]\right.}, \end{array}$$

where *N* is the total no. of observations and *C* is the total no. of classes. *P* represents the probability of observation *I* that belongs to class *c*.

## 4. Experimental Analysis and Findings

The proposed model used the train validate test approach. The model was fine-tuned using the validation data and then tested on the dataset. Since the dataset was large and the model needed repeatedly tuning parameters, the best approach was to split the dataset into three partitions. The data was split in the ratio of 70 : 15 : 15 for training, validation, and testing. The train validate split is shown in Table 2.

The data was trained on the model using 32 epochs with an Adam optimizer. It was observed that the training accuracy steadily kept increasing throughout all 32 epochs from 0.432 to 0.948. The validation accuracy, on the other hand, did not increase as smoothly. Validation accuracy for the first epoch was 0.61. Maximum validation accuracy achieved was 0.933, which stopped improving beyond epoch 25, as shown in Figure 5. The test accuracy was equal to 0.9113.

The training loss computed using categorical cross entropy was highest at 1.44 at the first epoch and steadily decreased at each epoch till it reached 0.14 at the last epoch. The validation loss did not decrease as smoothly and fluctuated quite a bit during epochs. It began at 1.04 and gradually declined. The loss fluctuated between 3.0 and 2.5 from epochs 16 to 31 and rose drastically to 0.40 in epoch 32, as shown in Figure 6.

Figure 7 is the confusion matrix of our model. For each class, the correctly classified and misclassified values can be seen. 113 out of 122 test images were classified accurately for the class dyskeratotic whereas nine cell images were misclassified. One hundred twelve cell images were correctly classified out of 124 test images for koilocytotic. Twelve cell images were misclassified. For the class, metaplastic 102 images were for the true class out of a total of 119 test images, and 17 images were not correctly classified. 115 out of 119 images were correctly classified for the parabasal class. Four test images were wrongly classified. Lastly, for the superficial-intermediate class, out of the 125 test images, 113 were correctly classified, and 12 were misclassified.

Results conclude that the proposed CNN model is computationally simple and does not require much time to train, validate, and test. It yielded a pretty good accuracy and had a low misclassification rate. The model performs poorly as the number of epochs exceeds 15. Fine-tuning the parameters will help overcome these shortcomings.

## 5. Conclusion

Cervical cells have complex anatomy and require hours and hours of physical examination in a laboratory setting to examine them. With the growth in the number of cervical cancer cases, it has become the need of the hour to not only diagnose cervical cancer in the precancerous or early stages but also reduce the overhead cost involved by reducing the time and resources spent during diagnosis. We used data from the publicly available cervical cell images dataset SIPaKMeD and trained a CNN model to classify cell images into five major cell categories. This classification enables health practitioners to distinguish normal cells from abnormal cells and predict precancerous cervical cell abnormalities. An 11-layer CNN architecture comprising four convolutional layers, three max-pooling layers, three dense layers, and one flatten layer has been used in the architecture. ReLU and sigmoid activation functions were used to achieve the desired results. Overall testing accuracy of 91.1% was achieved using this simple yet efficient model. Researchers can enhance this model to obtain faster results as promising as the computationally demanding AlexNet, VGGNet, and ResNet models employed in other recent research. For future improvements, the model should be trained on a bigger pool of Pap smear images to provide a better generalization.

## Figures and Tables

**Figure 1:** The proposed model workflow.

**Figure 2:** A koilocytotic cell.

**Figure 3:** A parabasal cell.

**Figure 4:** The proposed CNN architecture.

**Figure 5:** The training and test accuracy of the proposed model per epoch.

**Figure 6:** The training and testing loss of the proposed model per epoch.

**Figure 7:** Confusion matrix of the proposed model for the five cell categories.

**Table 1:** Data augmentation techniques applied to the dataset.

Data augmentation technique	Values
Zoom range	0.2
Sheer range	0.2
Rescale	1/255
Horizontal flip	True

**Table 2:** Train validate test split of the dataset.

Cell type	Total images	Train	Validate	Test
Dyskeratotic	813	569	122	122
Koilocytotic	825	577	124	124
Metaplastic	793	555	119	119
Parabasal	787	550	118	119
Superficial-intermediate	831	581	125	125

## Data Availability

The [Cervical Cancer Detection] data used to support the findings of this study are included within the article.
